# Virtual Reality-Based Analysis of Pressure Ulcer Care Information Related to Medical Equipment for the Prevention of Pressure Ulcer Skin Foam Dressings in the Elderly

**DOI:** 10.1155/2021/6389001

**Published:** 2021-11-09

**Authors:** Na Zhao, Zhanhong Tian, Yang Li, Haihua Yu, Yu Yang

**Affiliations:** ^1^Outpatient Dressing Room, Beijing Huairou Hospital, Huairou 101400, Beijing, China; ^2^Department of Respiration, Beijing Huairou Hospital, Huairou 101400, Beijing, China; ^3^Department of General Surgery, Beijing Chaoyang Hospital, Chaoyang 100015, Beijing, China; ^4^Department of Obstetrics and Gynecology, Beijing Huairou Hospital, Huairou 101400, Beijing, China; ^5^Department of Endocrine, Beijing Huairou Hospital, Huairou 101400, Beijing, China

## Abstract

As the standard of life has increased with the advancement of the time, there has been an increasing stress on healthcare with the aging diet, and pressure sores occur in elderly hospitalized subjects. Of course, the emergence of related medical devices, especially auxiliary foam dressings, is constantly improving. Pressure ulcers are extremely harmful to the elderly. The use of virtual reality technology to simulate the treatment of foam excipients is to test the role of medical devices in virtual reality. In particular, the use of foam dressings in the management of pressure deposits is the most relevant study for this paper, which reviews the relevant literature and conducts a thematic study on patients in a specific urban hospital. The relevant materials were designed, the experiments were designed, and the relevant research data were obtained. Studies show that virtual reality-based preventive medical devices can improve the efficiency of pressure ulcer treatment in hospitals by about 12%. Pressure ulcers have different incidences among people of different ages. The probability is much higher than that of adolescents. Foam dressing is very effective in preventing pressure ulcers. The probability of pressure ulcers after using foam dressing is about 35% lower than that when it is not used.

## 1. Introduction

As China's population ages and chronological diseases continue to advance, their danger is increasingly evident, with the elderly suffering the greatest portion of these illnesses. Meanwhile the trend of miniaturization of family composition and separation of two distinct generations has made the issue of empty nest elderly persons increasingly prominent. If not handled properly, this can create serious stress. Sores are a great threat to the health of the elderly. Meanwhile, with the promotion of an information and Internet of Things society, medical “smart” products are on the market [1]. As community education services and home care are increasingly broad in scope, the requirements are also expanding. For the time being, the pressure sore knowledge of community and home caregivers is missing or slow to be updated. Medical IoT can improve the correctness of data and extend the lifetime of network [2]. Because of the emergent and data-volumetric nature of data in healthcare IoT, the use of an event-driven approach is well suited for the monitoring of unexpected events [3]. As well, it allows nodes that are not located within the supervised regions to be in a slumbering state, decreasing the energy consumption of network ligatures [4].

Pressure sores occur in 3% to 12% of our inpatients, with a spectrum of the population being primarily elderly patients, with an incidence of 10% to 25% and a 6-fold improvement in the general population mortality rate, respectively, with statistics. The prevalence has not diminished compared to the preceding period. As the development of such pressure sores aggravates the physical and psychological pain of an individual patient, it has caused great economic loss; it increases the workload of nurses, gives rise to certain medical controversies, and takes up so many public health resources. It is one of the important issues requiring urgent solution in clinical nursing and is an important reference indicator for evaluating the quality of nursing care. A consensus has been reached globally that pressure sore preventing is the best treatment [5]. The frequency of intraoperative pressure sores in intracorporeal circulation surgery is as high as 16.7%, and they are highly valued by medical professionals [6].

On the issue of pressure ulcers, domestic and foreign experts are conducting some research on pressure ulcers. Xu Ting observes and analyzes approximately 10,000 patients and conducts controlled experiments on thousands of patients to observe the causes of pressure ulcers in hospitals and the differences between the two patient groups. Patients with pressure ulcers are treated according to preventive guidelines, observed for changes in pressure ulcer status after relevant precautions and relevant through experiments that standardize the relevant behavior of nurses in patient care [7, 8]. To investigate the causes of pressure ulcers, Yu Hui built a pressure ulcer prevention research model. By investigating inpatients, the feasibility of the model was validated and the characteristics of pressure ulcers in inpatients in my country were obtained. Through interviews with relevant healthcare professionals, the model was completed, patients within the model were categorized and analyzed, the reasons for the patient's pressure ulcers were identified, and targeted preventive suggestions were proposed for the relevant reasons. This is very powerful. For subsequent research, the reader is referred to [9].

This paper will provide a framework for the analysis of research and studies on this theme by organizing and classifying information obtained from literature research techniques and providing an analysis of medical Internet information. Designing a clinical trial to combine scientific research with empirical studies to investigate the causes of pressure sores and prevent them may increase the research on pressure sores by professionals involved with specialized research.

## 2. Analysis Method of Pressure Ulcer Care Information

### 2.1. Pressure Ulcers and Their Assessment

The most fundamental reason for pressure ulcers is that the body tissue is under pressure for a long time or is overcompressed, and impaired blood circulation in the local tissue causes ischemic hypoxic necrosis, which leads to the development of ulcers [10]. Due to the long operation time, the body's activity intensity during the operation is very low, the local tissue is compressed for a long time, and the hemodynamics are poor. In the case of improper nursing measures, it is easy to induce pressure sores. Reviewing a large number of literatures showed that the risk factors of intraoperative pressure ulcers include age, nutritional status, obesity, disease, smoking, surgical position, operation time, anesthesia, bleeding, intraoperative hypothermia, and hypotension [11, 12]. Many white blood cells that swallow and remove foreign substances are found in the local exudate, and the exudated fibrin gradually solidifies to form a protective barrier and prevent the invasion of bacterial toxins. This body's self-defense function can reduce infection to some extent. . It easily leads to pressure ulcers. Intraoperative anesthetic use relaxes skeletal muscles, causes loss of sensation, weakens muscle tone, temporarily loses protective response to physical discomfort, and causes pressure ulcers.

In the absence of knowledge about pressure sore prevention and treatment, chronically ill elderly patients are admitted with deep injuries, with varying degrees of infection, pronounced pain, and significant treatment durations [13, 14]. In this situation, the technique of topical dressing change is considered appropriate. Resident clinical patients agree with the drug change method and can cooperate actively with the procedure with high adherence [15]. In practice, it is necessary to conduct continuous evaluation and staged care for patients, pay attention to the effectiveness of special dressings, prevent the progression of pressure sores, and reduce the suffering of patients.

The most fundamental reason for pressure ulcers is that the body tissues are under pressure for a long time or excessively. The blood circulation disorder of the local tissues leads to ischemia and hypoxic necrosis, which leads to the occurrence of ulcers [16]. Due to the long operation time, the body's activity intensity during the operation is very low, the local tissue is compressed for a long time, and the hemodynamics are poor. In the case of improper nursing measures, it is easy to induce pressure sores. The prevalence of pressure ulcers during operation is related to the surgical position, and the surgical position determines the pressure position of the patient [17, 18]. Patients undergoing thoracoabdominal combined laparoscopic radical esophageal cancer surgery are first imaged in the left position and then in the supine position. Therefore, the patient's left ear, shoulder joint, left lateral chest, left ilium, lateral knee, and left outside of the ankle and the sacral coccyx are areas of pressure during the operation and are prone to pressure sores.

Correct assessment of the patient's condition is the key to preventing pressure ulcers during operation. Intraoperative pressure ulcers are different from ward pressure ulcers. During the entire operation, the nurse in the operating room plays a pivotal role in preventing pressure ulcers [19]. The pressure ulcer assessment scale used by operating room nurses to evaluate the risk factors of pressure ulcers is a key step in preventing pressure ulcers. Currently, the Waterlow assessment scale/Anderson assessment scale and Norton assessment scale are widely recognized and used in clinical work. However, in the current medical treatment, there are many and complicated risk factors for pressure ulcers in the operating room. Most of them are some attempts at improvement, and there is no reliability and validity test or lack of large sample clinical practice, and there is no standard operation [20].

Correct, safe, and rational surgical location is one of the key links to successful surgery and an important part of operating room risk management. While ensuring full exposure of the surgical field, it should be placed as much as possible in accordance with the patient's physiological structure to avoid damage to muscles and nerves [21]. In the operation of laparoscopic radical resection of esophageal cancer, it is necessary to change the position, first lying on the left side and then lying in the supine position. Therefore, itinerant nurses must master the standardized intraoperative placement of the left and supine positions and cooperate with the doctor to change the position. The surgical position includes the patient's position, the correct use of the posture cushion, and the operation of the operating table. Correct placement is the key to ensuring a reasonable and effective surgical position. The reasonable use of gel pads can make the patient evenly stressed and reduce local compression; and the safe operation of the operating table can prevent the body from being damaged by strong external forces. The surgical position is according to the lateral position operating specifications. The highest incidence of lateral pressure ulcers is in the axillary chest, which accounts for half of the pressure ulcers, with the anterior superior iliac spine and anesthesia sphygmomanometer cuff compressing the skin. At the place, the gel body cushion is composed of a base mask, a face mask, and an inner gel filling. It has a soft texture and good tissue compatibility. The gel solid has no fluidity. When placed, the body weight can be evenly distributed on the body cushion, reducing the local area. The pressure of the skin's hands and the use of gel pads instead of traditional sponge posture pads can better conform to the patient's body, reduce the pressure and shear force on the skin, effectively avoid the occurrence of pressure sores [22], and put a foam dressing on the bones of the upper spine, ankle and sacrum. The foam dressing is composed of an antiadhesion skin contact layer, a foam layer, and a waterproof and antibacterial top film, which can significantly reduce the friction between the skin and the operating bed and improve local blood and effectively prevent the occurrence of pressure sores.

Typical intraoperative pressure ulcers are primarily stage I and stage II pressure ulcers. These pressure ulcers first manifest as damage to muscle and subcutaneous tissue and then involve the dermis and epidermis and are more likely to occur in the carina of the bone. It takes 1-5 days to show obvious performance [23, 24]. Stage I and stage II pressure ulcers that appear immediately after surgery can rapidly develop into stage III and stage IV pressure ulcers within a few hours. This is why the intraoperative and 1 to 6 days after surgery are now related to the pressure ulcers of the surgical position. Pressure ulcers are called intraoperative pressure ulcers. Studies showed that all postoperative pressure ulcers appeared within 5 days postoperatively. Of these, 18.9% to 31% of patients may experience redness of the skin immediately after surgery, and 30% to 50% of these skin pressure ulcers develop into pressure ulcers.

### 2.2. Foam Dressing

Air-foam dressings improved leukocyte counts that were found in students with deep pressure lesions, a result that is in line with other researches. The hydrocolloid component of the foam dressing promotes autolytic wound debridement, limits inflammation, produces oxygen deficient tension, and sparks the release of macrophages and interleukins. It was shown that the use of camphor dressings instead of tracheostomy wound gown dressings in patients with stroke reduced the number of wound gown dressings and effectively diminished the rates of infection [25]. It was shown that the utilization of camphor wound dressing for stroke patients with tracheostomy wound dressing can reduce the frequency of wound dressing replacement and effectively reduce the percentage of contraction.

Changing process requires prompt removal of necrotic histories after wound infection is under control. The growth of new granulation tissue will otherwise be impaired. Debridement of wound healing enters the sarcomeres stage and epithelial crawling stage [26]. This promotes local blood distribution, activates tissue morphology, promotes transport of nutrients, strengthens cytokine activity, and results in the proliferation of a high number of fibroblasts, thus allowing the rapid establishment of tissue and the formation of capillary networks.

In the case of pressure sores, varying support devices may be substituted for different areas of the body. In the case of sacrococcygeal decubitus ulcers, the patient can be instructed to make a thick hollow sponge pad under the body. For pressure sores on the knees, a soft pillow can be placed between the feet, and, for pressure sores on the ankles, a rubber glove can be used to make something like a water pad under the feet. What these measures can do is preventing the wound from getting worse. Healthcare providers should develop a reasonable plan based on objective data on the patient's compression sore staging, wound condition, and nursing assessment [27].

### 2.3. Virtual Reality Algorithm

Adoption of virtual reality and the use of large data is going to be a major trend in the development of the future; however, it needs more time to be realized fully for the available medical prescription rules and the already existing message systems. Many challenges still exist in the technical and operational aspects of virtual reality, with capacity and performance issues, security restrictions, and other issues yet to be resolved.

#### 2.3.1. Logistic Regression Algorithm

The logistic regression algorithm is actually the simplest algorithm in a neural network and it consists of a damage control function, which is also called the linear leverage function. This function has a higher value as possible.

(1) $$\begin{array}{c} \text{net}=\sum_{i=0}^{n}w_{i}x_{i},\\ o=\sigma \left(\text{net}\right)=\frac{1}{1+e^{-\text{net}}},\\ f\left(x\right)=\text{sigmoid}\left(w^{T}x+b\right). \end{array}$$

Replace *z* with *θ*^*T*^*x* to get the model algorithm function:

(2) $$\begin{array}{c} h_{\theta }\left(x\right)=g\left(\theta^{T}x\right)=\frac{1}{1+e^{-\theta^{T}x}}. \end{array}$$

Over the whole composite feature, for example, sigmoid is a static feature with no additional arguments. Therefore it would be the only argument.

For the purpose of building the damage control function, we build it because we need to a criterion under which the best model for the training specimen is searched.

A policy filter function is

(3) $$\begin{array}{c} {\left(h_{\theta }\left(x_{i}\right)\right)}^{y_{i}}{\left(1-h_{\theta }\left(x_{i}\right)\right)}^{1-y_{i}}. \end{array}$$

The larger the value is, the better the model fits the sample. The formula is as follows:

(4) $$\begin{array}{c} P=\left\{\begin{array}{c} 1\\ \exp\left(-\frac{E\left(X_{new}\right)-E\left(xol\;d\right)}{T}\right) \end{array}\right.. \end{array}$$

The corresponding equation is

(5) $$\begin{array}{c} -di\;v\left(\frac{\nabla u}{\left|\nabla u\right|}\right)-\lambda \left(u_{0}-u\right)=0. \end{array}$$

The problem can be converted into an optimization one as a result of a function. Allow the difference error multiplier function to be

(6) $$\begin{array}{c} E\left(x,y\right)=di\;v\left(\frac{\nabla u}{\left|\nabla u\right|}\right)-\lambda \left(u-u_{0}\right). \end{array}$$

We can get

(7) $$\begin{array}{c} u\left(x,y\right)=N\left(u_{0}\left(x,y\right),w\right),\\ t\left(s\right)=\exp\left(-\int_{0}^{s}\kappa \left(t\right)dt\right). \end{array}$$

This allows us to see that

(8) $$\begin{array}{c} \partial =1-t\left(s\right)=1-\exp\left(-\int_{0}^{s}\kappa \left(t\right)dt\right). \end{array}$$

At this time, each individual in the offspring population corresponds to the amount of change in the initial solution.

(9) $$\begin{array}{c} \Delta Ek=fitness\left(x^{\prime }\right)-avgfitness. \end{array}$$

In the above equation, *fitness*(*x*′) is the fitness of the current individual and *avgfitness* is the average fitness. The acceptance probability Pk is calculated as follows:

(10) $$\begin{array}{c} P_{k}=\exp\left(\frac{-k\Delta E_{k}}{t_{k}}\right). \end{array}$$

The algorithm can quickly find the local optimal solution, but it lacks the overall ability to master the search space, and the search process is difficult to enter the most effective area, which makes the algorithm inefficient in the early global search. In addition, the algorithm is more sensitive to parameters, and the evolution speed is difficult to guarantee. The number of iterations of the algorithm running function and the termination condition of the algorithm can be adjusted according to the probability that a better solution can be searched for within a limited number of iteration steps. These can improve the global search performance of the algorithm to a certain extent.

## 3. Pressure Ulcer Nursing Information Analysis Experiment

### 3.1. The Purpose of the Experiment

The purpose of the experiment in this article is to comprehensively understand the current situation of pressure ulcer-related knowledge and clinical practice of clinical nurses in our province and their knowledge training needs and to find the gap between their clinical nursing practice and the latest knowledge and concepts, so as to better guide and standardize the clinical nursing practice of pressure ulcers, analyze its influencing factors to provide reference information for the management department to formulate relevant policies, and combine the survey results to have relevant knowledge of the prevention and treatment of pressure ulcers in various forms, content, and time. Clinical practice training is to explore the best training methods suitable for the current situation in our province to improve the theoretical level of pressure ulcer-related knowledge and clinical practice capabilities of clinical nurses in our province and then improve the level of nursing in our province in order to improve the prevention and management of pressure ulcers. It can help reduce the incidence of pressure ulcers.

### 3.2. Inclusion and Exclusion Criteria

#### 3.2.1. Inclusion Criteria

The inclusion criteria were as follows: ① no occurrence of pressure ulcer in all patients before the operation, ② no mental illness and age ≥60 years, ③ the operation time being more than 4 hours, ④ general anesthesia, and ⑤ patients undergoing elective surgery. The above conditions must be met at the same time.

#### 3.2.2. Exclusion Criteria

The exclusion criteria were as follows: ① patients suffering from diseases that affect the observation of the skin, ② patients with diabetes and severe complications, and ③ patients with impaired skin integrity.

### 3.3. Data Collection

The preoperative visit is to collect the general information of the patient by the roving nurse, such as gender, age, education level, work status, current residence, marital status, payment method, current smoking status, blood pressure status, combined disease status, and the patient's body mass index (BMI), record the number, incidence, stage, location, and so forth, and fill out the surgical patient's skin care record sheet. Pressure ulcers occur immediately after surgery, 6 hours after surgery, and 24 hours after surgery. The evaluation criteria are the latest pressure ulcers established by NRS.

### 3.4. Statistical Processing

This article uses statistical software SPSS 19.0. The research data in this article is expressed as *n* (%), and the *χ*2 test is used to compare between groups. When *P* < 0.05, it means that the difference between groups is statistically significant.

## 4. Analysis of Pressure Ulcer Nursing Experiment

### 4.1. Distribution of Patients

In order to understand the characteristics of the pressure ulcer population in this survey for statistical calculations, we conducted a classified survey of patients and collected statistics on patients according to factors such as age and gender. The specific data are shown in Table 1.

From Figure 1, we can see that the probability of pressure ulcers is different between different ages. The population with spontaneous cerebral artery dissection causing cerebral infarction is mainly distributed in middle-aged and elderly people, from 46 to 60 years of age, accounting for half of the population in this survey. Among the young and middle-aged people, the probability of pressure ulcers is the smallest, accounting for only about 20% of the total. This shows that the main population of pressure ulcers is the middle-aged and elderly population, and the related treatment methods should also be tilted towards the aspect. A public view as to the cause of an induration has not emerged yet . A survey of patients was conducted to establish the causes of pressure sores by ascertaining the unusual physical factors that distinguish their body characteristics from those of the normal population where pressure sores happen. For details, see Table 2.

From Table 2, we can see that when a patient has a pressure ulcer, the patient's body temperature, pulse, and other data are all abnormal. The difference between patients is relatively large. The overall *P* value is less than 0.05, which is not statistically significant. We compare the vasoactive drugs, bleeding volume, and positioning time between patients, as shown in Table 3.

From Table 3, we can see that the difference between patients is not statistically significant. The intraoperative blood loss in the control group was 32.65 ± 8.25 (ml), and the intraoperative blood loss in the intervention group was 35.42 ± 9.42 (ml). After *t*-test, *P* = 0.111, and the difference is not statistically significant. After the *t*-test, the total time of operation and total time of posture placement showed that the difference between the two groups of patients was statistically significant.

### 4.2. Treatment Methods

According to medical standards, pressure ulcers can be divided into 4 stages of pressure ulcers. Each type of pressure ulcer is different according to its severity and related treatment options. The classification of pressure ulcers is shown in Figure 2 and Figure 3.

The current treatment for compression sores includes regular postural alterations, there is special pressure reduction on the mattress, and there is sufficient access to nutrition, antibiotics, and the foam dressing used here. We collected data on the current statistics of the population undergoing treatment. More detailed statistics are shown in Table 4.

As shown in Figure 4, when a patient develops a pressure ulcer, the pressure ulcer will be treated. However, because the treatment method has not been popularized, using the foam dressing studied in this article is not the first choice of the patient, and most patients still use it. The original experience is to prevent patients with such primitive methods as turning over frequently.

### 4.3. Therapeutic Effect

For patients suffering from pressure ulcers, the treatment effect of pressure ulcers has attracted much attention. Therefore, we have calculated the pressure ulcer treatment effect of patients under different prevention and treatment methods and digitized it through the model designed in this article. The specific data are shown in Table 5.

As shown in Figure 5, in this investigation, different methods of preventing and treating pressure ulcers can achieve certain results in practice, but, overall, the method of using foam dressings is in the process of treating and preventing pressure ulcers. Its various parameters are due to other methods, and the branch of the foam dressing must be about 0.8, which is excellent. It also shows the important role foam dressing could play in the prevention of decubitus ulcers. Prognostic care of pressure ulcers was also critically important. In this regard, some important signs of the prognosis were statistically calculated, which are shown in Table 6.

Figure 6 shows that, after treatment with different methods, the prognostic effect of each method is different. Overall, the use of foam dressings in this article has the best prognostic effect, with an average prognostic effect of about 0.8. The average value of other methods is about over 0.6. The authors show that foam dressing can play an important role in the prevention of pressure ulcers.

## 5. Conclusion

Flexible, elastic, and absorbent foam is composed mainly of polyvinyl alcohol foam and urethane. Most of the components of foam dressing are soft silicone mucilage, the special polymeric material made of water, oil, and silicon. They are nonstimulating to skin contact and flexible and have a certain thickness to the dressings to reduce discomfort and pain from local strain. From multiple perspectives and multiple specialties, we will jointly solve professional nursing problems such as the prevention and treatment of pressure ulcers in critically ill patients and, at the same time, help patients transfer out of the ICU as soon as possible, improve the professional care capabilities of critically ill patients, jointly provide patients with safe, reliable, and effective nursing services, reduce complications and mortality, improve the quality of clinical care, establish and improve the reporting system, report high-risk patients in a timely manner, and standardize pressure ulcer management. At the same time, hospitals need to develop or improve the “unavoidable pressure ulcer” system according to their specific conditions and characteristics and gradually establish a relatively complete system. Due to the limited conditions, the research in this article has only achieved results in the application of the first hospital in this city and has not conducted a multicenter large sample comparative study. The results are relatively limited. It needs to be promoted and applied in other specialized fields, and the sample size should be increased for further verification.

## Figures and Tables

**Figure 1:** Distribution of patients.

**Figure 2:** Different types of pressure ulcers.

**Figure 3:** Effect picture of pressure sore.

**Figure 4:** Number of people with pressure ulcers treated by different methods.

**Figure 5:** Treatment effect of different methods.

**Figure 6:** Prognostic treatment score.

**Table 1:** Distribution of patients.

	Vertical pressure	Friction	Shear force	Partial loss of moisture	Malnutrition	Other illnesses
0–12	13	8	11	7	8	2
13–26	6	8	3	4	1	4
27–45	7	6	9	16	6	7
46–60	30	21	17	15	13	9
Over 60	37	42	51	21	19	15

**Table 2:** Patient index comparison.

	Intervention group	Control group	Normal person	*T*	*P*
Body temperature	36.31 ± 0.36	36.53 ± 0.22	37.23 ± 0.22	−0.448	0.454
Pulse	71.48 ± 7.29	71.38 ± 7.02	72.26 ± 7.12	0.883	0.379
Breathe	12.78 ± 2.08	12.32 ± 1.82	13.12 ± 1.82	1.352	0.179
SpO_2_ (%)	92.24 ± 0.80	91.86 ± 1.68	91.96 ± 1.74	1.659	0.100
NRS	2.08 ± 0.35	1.98 ± 0.42	2.12 ± 0.62	1.052	0.295

**Table 3:** Comparison of intraoperative conditions of patients.

	Intervention group	Control group	Normal person	*T*	*P*
Bleeding volume	32.65 ± 8.25	35.42 ± 9.42	36.13 ± 0.12	−1.602	0.111
Total operation time	5.95 ± 0.85	5.95 ± 0.85	7.16 ± 0.52	−2.342	0.021
Total time of posture	22.42 ± 3.51	23.84 ± 4.08	23.72 ± 3.82	−2.143	0.034

**Table 4:** Treatment methods.

	Regular posture changes	Special mattress decompression	Adequate nutrient intake	Antibiotics	Foam dressing
Stage I pressure ulcer	13	29	47	31	21
Stage II pressure ulcer	9	21	51	26	13
Stage III pressure ulcer	6	54	23	47	29
Stage IV pressure ulcer	5	19	27	29	35
Nonstage pressure ulcers	2	16	19	26	32

**Table 5:** Treatment effect of radius fracture.

	Stability	High fever	Swelling of the skin	Pain	Wound healing	Treatment costs
Regular posture changes	0.537	0.887	0.528	0.718	0.642	0.516
Special mattress decompression	0.431	0.573	0.431	0.752	0.669	0.678
Adequate nutrient intake	0.479	0.526	0.888	0.697	0.477	0.617
Antibiotics	0.539	0.643	0.542	0.573	0.681	0.854
Foam dressing	0.879	0.735	0.779	0.727	0.813	0.595

**Table 6:** Prognostic care effect.

	Stability	High fever	Swelling of the skin	Pain	Wound healing	Treatment costs
Regular posture changes	0.478	0.817	0.559	0.697	0.679	0.542
Special mattress decompression	0.431	0.573	0.431	0.752	0.669	0.678
Adequate nutrient intake	0.479	0.526	0.823	0.697	0.435	0.617
Antibiotics	0.539	0.643	0.556	0.573	0.681	0.854
Foam dressing	0.842	0.798	0.697	0.735	0.826	0.789

## Data Availability

No data were used to support this study.
